The article "Chaiqin Qingning Capsule Inhibits Influenza Virus Infection and Inflammation In Vitro and In Vivo" was published in 2021. Journal: Evid Based Complement Alternat Med.

# Chaiqin Qingning Capsule Inhibits Influenza Virus Infection and Inflammation *In Vitro* and *In Vivo*

**DOI:** 10.1155/2021/6640731

**Published:** 2021-09-11

**Authors:** Jin Zhao, Yanbing Hao, Xuanzi Xia, Runfeng Li, Xiaodong Huang, Zifeng Yang, Xinhua Wang

**Affiliations:** ^1^State Key Laboratory of Respiratory Disease, National Clinical Research Center for Respiratory Disease, Guangzhou Institute of Respiratory Health, The First Affiliated Hospital of Guangzhou Medical University, Guangzhou Medical University, Guangzhou, Guangdong, China; ^2^Shantou University Mental Health Center, Shantou, China; ^3^Institute of Integration of Traditional and Western Medicine, Guangzhou Medical University, Guangzhou, China

## Abstract

**Background:**

Chaiqin Qingning Capsule (CQ-C) is a traditional Chinese medicine (TCM) formula commonly used to treat respiratory infectious diseases in China. The aim of this study was to detect the effect and mechanism of CQ-C treated with influenza virus *in vitro* and *vivo*.

**Methods:**

The cytotoxicity and antiviral activity of CQ-C *in vitro* was determined by methyl thiazolyl tetrazolium (MTT) assay. The regulation of CQ-C on cytokine/chemokine expression was evaluated using RT-qPCR. In addition, the effect of CQ-C on the pathway protein, NF-*κ*B, and its phosphorylation level was verified by western blotting. After virus inoculation, BALB/c mice were administered with CQ-C of different concentrations for 7 days. Body weight, viral titer, lung pathology, and mortality of the mice were measured, and the level of inflammatory cytokines was also examined using real-time RT-qPCR.

**Results:**

CQ-C inhibited the proliferation of influenza virus of various strains *in vitro*, with the 50% inhibitory concentration (IC50) ranging from 49 to 59 *µ*g/mL. CQ-C downregulated virus-induced gene expression of IL-6, TNF-*α*, CXCL8, CXCL10, CCL5, and COX-2 in a dose-dependent manner in A549 cells. Also, CQ-C inhibited the expression of NF-*κ*B protein of the signaling pathway. Moreover, a decrease of the lung index and mortality of mice was observed in the CQ-C (1 g/kg/d) group. The related cytokine/chemokine expression was also decreased in the early stages of infection in the mRNA level.

**Conclusion:**

As a clinically applied Chinese prescription, our study shows that CQ-C has a wide range of effects on several influenza viruses. Moreover, CQ-C could play an important role in anti-influenza activity and anti-inflammation *in vitro* and *in vivo*. Thus, CQ-C may be a promising treatment option for influenza.

## 1. Introduction

Influenza is an infectious disease that seriously affects human life and health. Influenza virus is a common respiratory pathogen, which occurs globally with an annual attack rate estimated about 3 to 5 million cases of severe illness and about 250,000 to 500,000 death [1]. Especially, the 1918–1919 influenza pandemic caused an estimated 50 million deaths [2, 3]. Similar to the 1918 pandemic, the 2009 influenza A virus pandemic caused more severe and fatal cases among people aged 30-50, which constituted up to one-third of patients in hospital [4, 5]. More recently, other influenza viruses (including H5N1, H5N6, and H5N8) have emerged and posed serious threats to public health [6].

It is well known that the virus not only replicates but also can cause strong inflammatory response, which contributes to sever diseases or death. Influenza virus is firstly recognized by the innate immune system through pattern recognition receptors (PRRs), such as the toll-like receptors, retinoic acid-inducible gene I, and nucleotide-binding oligomerization domain- (NOD-) like receptors, which leads to the production of type I interferons (IFNs), proinflammatory cytokines, eicosanoids, and chemokines [7]. Moreover, virus-induced high levels of cytokines could result in the development of acute respiratory distress syndrome (ARDS) [8], which also was observed in COVID-19 patients [9]. Thus, excessive activation of monocyte/macrophage and proinflammatory cytokines and chemokines causing cytokine storms contributes to acute lung immunopathology and the severity of the disease [10]. These studies suggested that inhibiting immune response disorder may provide the therapeutic benefit during influenza virus infection [11, 12].

Antiviral drugs were widely used in inhibiting influenza virus replication and inflammation response in clinical trials. At present, there are several therapeutic drugs for influenza virus, such as oseltamivir, zanamivir, and peramivir; however, they have some side effects and drug resistance [13]. Therefore, the development of new antiviral drugs as alternative therapies may be urgently needed.

Traditional Chinese medicines have been used to treat infectious diseases for thousands of years in China. Recently, several types of these herbal medicines have been used for treatment of influenza infection [14–18]. Chaiqin Qingning Capsule (CQ-C), which composed of baicalin (*Scutellaria baicalensis* Georgi.), Radix Bupleuri extract (*Bupleurum chinense* DC.) and Calculus Bovis Artifactus (Rengong niuhuang), has been used commonly for the treatment of cough, cold, fever, headache, bronchitis, sore throats, nasal congestion, and chronic bronchitis [19–22]. In addition, the CQ-C, including some of its components, has been already used in animal experiment because of its reasonable dose and effect [19, 22]. Although baicalin and saikoside A have been reported to have anti-influenza virus effect [21, 22], however, the treatment and prevention of H1N1(A/PR8/34) virus strain (PR8) infection with CQ-C have not been investigated. Therefore, to further explore the protective mechanism of CQ-Cagainst influenza virus, the antiviral effect and inmmunomodulatory potential of CQ-C *in vivo* and *in vitro* were investigated.

## 2. Methods

### 2.1. Chemicals and Reagents

Human alveolar epithelial cell line (A549) and Madin–Darby Canine Kidney (MDCK) cells were purchased from ATCC. These cells were propagated at 37°C under 5% CO_2_ in Dulbecco's Modified Eagle's Medium (DMEM) or Modified Eagle Medium (MEM) supplemented with 10% fetal bovine serum, 100 U/mL penicillin, and streptomycin.

Influenza virus A/PR/8/34(H1N1), A/Guangzhou/GIRD07/2009 (H1N1), A/HK/8/68(H3N2), A/HK/Y280/97 (A/H9N2), and B/Lee/1940 (FluB) were used in this study. Virus stocks were prepared in the allantoic cavities of chicken eggs, and aliquots were stored at −80°C. Virus titers were determined by 50% tissue culture infectious dose (TCID_50_) assay in confluent MDCK cells in 96-well plates. MTT was purchased from Sigma-Aldrich Chemicals Co. (St. Louis, MO, USA).

### 2.2. Preparation and Component Identification of CQ-C

The CQ-C extract was prepared by the Yangtze River Pharmaceutical Group, Jiangsu, China. In a previous study, a high-performance liquid chromatography-miangsuass spectrometry/MS (HPLC-MS/MS) method was employed to detect ten bioactive components for the quality control of CQ-C [23]. HPLC-MS/MS revealed that CQ-C contained baicalin, cholic acid, taurocholic acid, deoxycholic acid, hyodeoxycholic acid, chenodeoxycholic acid, saikosaponin A, saikosaponin B1, saikosaponin C, and saikosaponin D [23]. Radix Bupleuri (1000 g) was extracted in 60% ethanol at room temperature for 3 days; after filtration, the gruffs were also extracted in 60% ethanol for 3 days ethanol. The two extracts were collected and concentrated under reduced pressure to the relative density of 1.20∼1.25 (50∼55°C). Then, the three component herbs of CQ-C were admixed in the prescribed proportion (%, w/w) (Table 1).

### 2.3. Cell Cytotoxicity Assay

The 50% cytotoxic concentration (CC_50_) of CQ-C extract on MDCK and A549 cells was assayed using an MTT assay. The serial dilutions of CQ-C extract for the cytotoxicity assay were 1000, 500, 250, 125, 62.5, 31.25, 15.625, and 7.8125 *µ*g/mL. The CC_50_ was calculated using regression analysis.

### 2.4. Inhibition Assay of CQ-C

MDCK cells were grown in 96-wells plates (5 × 10^4^ cells per well) at 37°C for 24 h. The medium was replaced with a serum-free medium (100 *μ*L/well) containing 100TCID_50_ virus and various concentrations of drugs. After 2 h of incubation, the culture supernatant was removed and the cells were washed three times with phosphate buffered saline (PBS) and the cells were cultured with MEM. After 48 h incubation, the viability of cells was determined by MTT assays. The half maximal effective concentration (EC_50_) was calculated using regression analysis.

### 2.5. Real-Time Quantitative PCR Analysis

The relative gene expression in A549 cells or mice infected with A/PR/8/34(H1N1) was analyzed using RT-qPCR. Total RNA was extracted with 1 ml of TRIzol™ reagent (Invitrogen Life Technologies). cDNA reaction employed the PrimeScript RT-PCR Kit (Takara Bio). RT-qPCR was performed and analyzed by using an ABI7500 system (Applied Biosystems) as previously described [24]. Forward and reverse primer sequences for IL-6, TNF-*α*, CXCL8, CXCL10, CCL5, COX-2, and GADPH genes were designed on the PubMed website(Table 2). Relative gene expression levels were calculated as 2^−△△CT^ [25, 26].

### 2.6. Western Blotting

A549 cells were infected with PR8 (MOI = 0.2) at 2 h.p.i. and then switched to a serum-free medium or CQ-C (100, 50, 25, and 12.5 *µ*g/mL) in each group for 48 h and harvested for western blot analysis. The total proteins of the samples were extracted from the cells with radioimmunoprecipitation assay (RIPA) buffer (DGCS Biotechnology, China). The protein concentrations of each group were detected by using the BCA kit (Beyotime, China). Then, 15 ng of the cell extract was separated by 8% sodium dodecyl sulfate polyacrylamide gel electrophoresis (SDS-PAGE), and then, they were transferred to a polyvinylidene fluoride (PVDF) membrane (Millipore, USA). The membranes were blocked with 5% BSA at room temperature for 2 h and incubated with NF-*κ*B, rabbit monoclonal (Signaling Technology, Inc., Lot No: 8242), and p-NF-*κ*B rabbit monoclonal (Cell Signaling Technology, Inc., Lot No: 3033) antibodies overnight at 4°C. Then, the membranes were incubated with secondary antibodies for 1 h. Proteins were visualized by incubating membranes with Pierce enhanced chemiluminescence (ECL) plus western blotting substrate (Thermo Scientific), followed by detection on Syngene PXi9-TCH Access.

### 2.7. Protective Effect of CQ-C in Mice

Specific-pathogen-free BALB/c female mice weighing approximately 14 to 16 g were purchased from the Guangdong Medical Laboratory Animal Center (Guangzhou, China). The animal research was performed in the ABSL-2 Laboratory of the First Affiliated Hospital of Guangzhou Medical University. This study was approved by the Ethics Committee of the First Affiliated Hospital of Guangzhou Medical University (No. 2020224).

Mice were randomly divided into the control, virus-infected CQ-C, and Oseltamivir (OSE) treatment groups (10 mice per group). After anesthetized with isofurane, mice were infected with influenza virus A/PR/8/34(H1N1) (mouse adapted) intranasally at 2 LD_50_ (50% lethal dose) of dosage in a volume of 50 *μ*L per mouse. The daily dosage of CQ-C was translated from the clinical dosage of adult human (60 kg) using a previously described formula [27]. Also, the initial drug treatment（CQ-C） was administered 2 days before virus challenge. Then, the inoculated mice received different concentrations of CQ-C extract (1 g/kg/d or 500 mg/kg/d, dissolved in saline), oseltamivir (60 mg/kg/d, dissolved in saline), or saline twice daily for 5 days. The survival of mice was monitored until 14 d.p.i.

### 2.8. Lung Viral Titer, Lung Index, and Histopathological Change Detection in Mice Infected with H1N1

For lung virus titer determination, 5 mice from each group were euthanized at 5 d.p.i (day postinfection) and the lung tissues were harvested. The lung samples were homogenized in the MEM containing antibiotics (0.1% penicillin-streptomycin), centrifuged at 12,000 rpm for 10 min at 4°C, and stored at −80°C for further analysis. The lung homogenate supernatant was determined according to the virus titer using end-point titration in MDCK cells. Also, they also were determined for inflammatory cytokines and chemokine expression (gene sequence shown in Table 3) by using real-time RT-qPCR as previously described [25]. For lung index and the lung lesion assay, 5 mice from each group were euthanized by euthanasia at 5 d.p.i. and the lung tissues were harvested and weighed. Then, the lung tissues were fixed with 10% formaldehyde solution and were subjected to standard hematoxylin and eosin staining detection [28].

### 2.9. Statistical Analysis

Data are presented as the Mean ± SD. All data were analyzed using GraphPad and SPSS 17.0 software. Weight data were checked by repeated measurements and a mixed model multivariate analysis of variance. Statistics were analyzed with ANOVA or two-tailed Student's t-test. The probability of mouse survival was estimated by the Kaplan–Meier method. Statistical significance was set as *P* < 0.05.

## 3. Results

### 3.1. CQ-C Extract Inhibits Influenza Virus Replication in MDCK Cells

Firstly, the cytotoxic effect of CQ-C extract was detected using an MTT assay. The CC_50_ of CQ-C extract towards MDCK and A549 cells was 130.14 and 195.45 *µ*g/mL, respectively. In addition, the antiviral effect of CQ-C extract was investigated in cultured cells. Also, the results showed that CQ-C could significantly inhibit several influenza viruses, such as A/PR/8/34(H1N1), A/GZ/GIRD07/09(H1N1), and A/HK/8/68(H3N2), as shown in Table 4. CQ-C extract exhibited inhibitory activities, with IC_50_ ranging from 48.98 to 59.05 *μ*g/mL and a selective index (SI) ranging from 2.20 to 2.66. However, CQ-C displayed no effect towards B/Lee/1940 and avian influenza virus A/HK/Y280/97(A/H9N2).

### 3.2. CQ-C Extract Inhibits Influenza A Virus-Induced Cytokine/Chemokine Expression in A549 Cells

To examine the inhibition effect of CQ-C on virus-induced inflammatory responses, influenza virus-induced expression of cytokine/chemokine in A549 cells at 24 h after infection was measured using RT-qPCR. Virus infection induced a robust increase of IL-6, CXCL8, TNF-*α*, CXCL10, COX-2, and RANTES in mRNA level with a dose-dependent manner (Figure 1).

### 3.3. Effect of CQ-C on Proteins of the NF-*κ*B Signaling Pathway

The NF-*κ*B signaling pathway is important for efficient influenza A virus growth. To further study the underlying anti-inflammation mechanisms of CQ-C, the NF-*κ*B signaling pathway-related proteins were determined by western blotting. The protein expression of p-NF-*κ*B, NF-*κ*B contrast to GAPDH in the CQ-C-treated groups and virus group or control group is shown in Figure 2. Compared to the virus group, the expression of the p-NF-*κ*B was slightly reduced in A549 cells compared with that of the CQ-C group (100 *μ*g/mL), while the expression of p-NF-*κ*B in the CQ-C groups (50, 25 *μ*g/mL) was not significantly different.

### 3.4. Effects of CQ-C on Mice

The symptoms of ruffled fur, lethargy, and reduced food intake 4 days after infection were observed in mice infected intranasally with influenza virus. The lethal infection appeared in several animals at 6 d.p.i. After day 11, no additional animals died, and the survival rate remained stable in each group. The survival rates of the CQ-C (1 g/kg/d, 500 g/kg/d)-treated groups on 14th d.p.i were 100.0% and 50.0%, which are higher than those of the viral group (30.0%) (Figure 3(a)). These results demonstrate that CQ-C could prevent influenza virus-induced death in mice.

The body weight of the mice in each group was also measured. Administration of CQ-C extract (1 g/kg/d) effectively protected the infected mice from weight loss caused by influenza virus infection (Figure 3(b)). Animals treated with CQ-C extract at 1 g/kg/d recovered weight starting on day 9, in spite of a similar trend of initial weight loss in the first 7 days. These results manifested that treatment with CQ-C could improve weight loss of mice and decrease the mortality. CQ-C also had a tendency to decrease lung index causing by influenza virus, but there was no statistical significance (Figure 3(c)),and it also did not decrease virus titration at 5th d.p.i (Figure 3(d)). Viral pneumonia was the main pathological damage in the mice infected with influenza virus [27, 29]. Our study also observed these pathological changes on day 5th after virus inoculation. Lung tissue of infected mice showed epithelial cells apoptosis, infiltration of monocytes and lymphocytes, thickened alveolar walls, and exudation of inflammatory cells into the alveolar space, whereas treatment with CQ-C ameliorated and improved the pathological injury in a dose-dependent manner (Figure 4). Taken together, our results suggest that the CQ-C extract can efficiently protect mice from influenza virus infection and alleviate the lung lesions.

To determine the immune regulatory effect of CQ-C, lung tissues were collected at 4 d.p.i and then the cytokines were detected and analyzed. Treatment with CQ-C (1 g/kg/d) showed the expression of TNF-*α*, as well as chemokines (CXCL9 and CXCL10) were reduced clearly, compared with those from influenza virus-infected mice, as shown in Figure 5.

## 4. Discussion

Influenza virus can cause the flu, threaten the health of humans, and kill several thousand people every year worldwide [1]. Despite the development of antiviral drugs, the occurrence of drug-resistant viruses and side effects of the drugs are still frequently reported [30]. Therefore, safe and effective antiviral agents are urgently needed. Nowadays, the traditional Chinese medicines are widely used as antivirus agents by inhibiting the replication of influenza virus directly and improving the immune functions of the host organism [24, 31–33]. CQ-C, as a TCM formula, has the advantage of safety and small side effects [22], compared with some anti-influenza drugs or combinations of agents, such as oseltamivir and amantadine [34, 35]. Our results showed that the CQ-C inhibited several influenza viruses and decreased the expression of some of inflammatory cytokines induced by influenza virus and also can exert the influence on the NF-*к*B signaling pathway.

In this study, we found that the CQ-C could inhibit several influenza viruses and reveal an effective antiviral capacity, which suggested CQ-C had a certain range inhibitory effect on common respiratory viruses. However, it has no effect on avian influenza and hand-foot-mouth disease-related enterovirus. As is well known, influenza virus infection induces host innate immune responses, which results in virus replication, and meanwhile, abnormal proinflammatory innate immune responses correlate with increased morbidity and mortality [7]. Previous studies have shown influenza infection can cause the production of TNF-*α*, IL-1*β*, IFN-*γ*, and IL-6 [27, 36–38]. So, in the present study, we demonstrated that the CQ-C decreases the expression of IL-6, TNF-*α*, CXCL8, CXCL10, CCL5, and COX-2 induced by influenza virus in a dose-dependent manner (Figure 1). These results indicated that CQ-C has a better effect on the inflammation response induced by influenza virus.

The NF-*κ*B signaling pathway activation induced by virus infection has been proved to play an important role in regulating inflammation responses and other cellular activities [39, 40]. Our data showed that CQ-C (100 *µ*g/mL) induced the expression of p-NF-*к*B protein and regulated the levels of NF-*к*B phosphorylation. It is expected that CQ-C exerts protective effects against the inflammatory response in the process of influenza virus infection.

To further study the antiviral effect of influenza virus *in vivo*, the antiviral and anti-inflammatory activity of CQ-C in mice infected by influenza virus were detected. Our results showed that mice infected with PR8 at 2 LD_50_ of dosage could manifest viral pneumonia. Treating with CQ-C (1 g/kg/d and 500 mg/kg/d) could the increase survival rate and improve lung pathological damage and lung index. It was found that oseltamivir had a much better inhibitory effect on the virus titer of lung tissues than that of CQ-C. However, the production of cytokines/chemokines (TNF-*α*, CXCL9, and CXCL10) were significantly decreased in the CQ-C group (at 4 d.p.i), compared with the virus group, and moreover, QC-C has similar anti-inflammatory effects, compared to oseltamivir, which indicated that CQ-C accelerated recovery from infection in mice and might improve the immune environment of the mice. Therefore, CQ-C may be an effective anti-influenza drug via improving lung inflammatory response and lung tissue lesions.

## 5. Conclusions

As a clinically applied Chinese prescription, our study shows that CQ-C manifests a wide range of effects on several influenza viruses. Moreover, CQ-C could play an important role in anti-influenza (H1N1/PR8) activity and anti-inflammation *in vitro* and *in vivo*. Thus, CQ-C may be a promising treatment option for influenza.

## Figures and Tables

**Figure 1:** Effect of CQ-C on mRNA expression of cytokines/chemokines in A549 cells induced by influenza virus. A549 cells infected with A/PR/8/34(H1N1) (MOI = 0.2) were treated with CQ-C (50–100 *μ*g/mL) for 24 h prior to extract RNA. The mRNA level of cytokine/chemokine (IL-6, TNF-*α*, CXCL8, CXCL10, CCL5, and COX-2) was analyzed using RT-qPCR, ^*∗*^*p* < 0.05, ^*∗∗*^*p* < 0.01, and ^*∗∗∗*^*p* < 0.001,when compared with the virus group.

**Figure 2:** The expression of the NF-*κ*B and p-NF-*κ*B proteins in the A549 cells was detected by western blot analysis.

**Figure 3:** The protective activities of CQ-C on lethal influenza virus-infected mice *in vivo*. (a) The survival curve for indicated groups (*n* = 10 per group); (b) changes in body weight after infection. Mice were intranasally infected with 2LD50 and monitored for changes in body weight daily for 14 days (*n* = 10 per group); (c) organs index. Mice were sacrificed to calculate lung index, spleen index, and thymus index on day 5 after infection (*n* = 5 per group); and (d) lung virus titer (*n* = 5 per group); ^*∗∗*^*p* < 0.01 and ^*∗*^*p* < 0.05, when compared to the control group.

**Figure 4:** Histological observations of lung tissues for mice sacrificed at the 5th d.p.i. (a), (b) Influenza virus-infected mice treated with 1000 or 500 mg/kg/d of CQ-C (100X magnification). (c) Influenza virus-infected mice treated with 60 mg/kg/d of oseltamivir; (d) mock-infected mice treated with PBS (normal control, NC); and (e) influenza virus-infected mice treated with PBS (viral control, VC).

**Figure 5:** The level of cytokines CXCL9, CXCL10, and TNF-*α*. Mice per groups were sacrificed to determine the level of cytokines by RT-qPCR at day 4 after infection. ^*∗*^*p* < 0.05 and ^*∗∗*^*p* < 0.01, when compared with the virus group.

**Table 1:** Component herbs and typical active ingredients of CQ-C.

Pharmaceutical name	Composition (% w/w)
Baicalin	32.6
Bupleurum	36.4
Calculus bovis	31

**Table 2:** Human primers and probe sequences for qRT-PCR.

Gene	Primers and probe	Sequence (5'-3')
CXCL8	Forward	TTGGCAGCCTTCCTGATTTC
	Reverse	TATGCACTGACATCTAAGTTCTTTAGCA

CXCL10	Forward	GAAATTATTCCTGCAAGCCAATTT
	Reverse	GAAATTATTCCTGCAAGCCAATTT

CCL5	Forward	CAGCAGTCGTCTTTGTCACC
	Reverse	GTTGATGTACTCCCGAACCC

TNF-*α*	Forward	AACATCCAACCTTCCCAAACG
	Reverse	GACCCTAAGCCCCCAATTCTC

IL-6	Forward	CGGGAACGAAAGAGAAGCTCTA
	Reverse	CGCTTGTGGAGAAGGAGTTCA

COX-2	Forward	GAATCATTCACCAGGCAAATTG
	Reverse	TTTCTGTACTGCGGGTGGAAC

GADPH	Forward	GAAGGTGAAGGTCGGAGTC
	Reverse	GAAGATGGTGATGGGATTTC

**Table 3:** Mouse primers sequences for qRT-PCR.

Gene	Primers and probe	Sequence (5'-3')
CXCL9	Forward	TCTTGCTGGTTCTGATTGGAGT
	Reverse	GATAGTCCCTTGGTTGGTGCTG

CXCL10	Forward	GAAATTATTCCTGCAAGCCAATTT
	Reverse	TCACCCTTCTTTTTCAT-TGTAGCA

TNF-*α*	Forward	AACATCCAACCTTCCCAAACG
	Reverse	GACCCTAAGCCCCCAATTCTC

GADPH	Forward	GAAGGTGAAGGTCGGAGTC
	Reverse	GAAGATGGTGATGGGATTTC

**Table 4:** Inhibitory effects of CQ-C against influenza virus *in vitro*.

Virus strains	TC_50_	IC_50_	SI
A/PR/8/34(H1N1)	130.14	59.05 ± 0.13	2.20
A/GZ/GIRD07/09(H1N1)	130.14	56.87 ± 0.59	2.29
A/HK/8/68(H3N2)	130.14	48.98 ± 0.33	2.66
A/HK/Y280/97(H9N2)	130.14	>131	<1
B/Lee/1940(FluB)	130.14	>131	<1

## Data Availability

The data used and/or analyzed during the current study are available in this published article and from the corresponding author on reasonable request.

## Abbreviations

ARDS: Acute respiratory distress syndrome
CC50: 50% cytotoxicity concentration
CQ-C: Chaiqin Qingning Capsule
d.p.i: Day postinfection
ECL: Enhanced chemiluminescence
IC50: The 50% inhibitory concentration
IFNs: Type I interferons
MDCK: Madin–Darby Canine Kidney
TCM: Traditional Chinese medicine
MTT: Methyl thiazolyl tetrazolium
MEM: Modified Eagle Medium
NOD: Nucleotide-binding oligomerization domain
PBS: Phosphate buffered saline
PRRs: Pattern recognition receptors
PVDF: Polyvinylidene fluoride
RIPA: Radioimmunoprecipitation assay
TCID50: 50% tissue culture infectious dose
WHO: World Health Organization.
